The article "Stereotactic radiosurgery combined with anlotinib for limited brain metastases with perilesional edema in non‐small cell lung cancer: Rvision‐001 study protocol" was published in 2020. Journal: Thorac Cancer.

# Stereotactic radiosurgery combined with anlotinib for limited brain metastases with perilesional edema in non‐small cell lung cancer: Rvision‐001 study protocol

**DOI:** 10.1111/1759-7714.13386

**Published:** 2020-03-12

**Authors:** Yuxia Wang, Xin Wang, Yun Guan, Yongchun Song, Hongqing Zhuang, Enmin Wang

**Affiliations:** ^1^ Department of Radiation Oncology Peking University Third Hospital Beijing China; ^2^ Department of Neurosurgery, Huashan Hospital Fudan University Shanghai China; ^3^ Department of Radiotherapy Tianjin Medical University Cancer Institute and Hospital, National Clinical Research Center for Cancer, Key laboratory of Cancer Prevention and Therapy Tianjin China

**Keywords:** Anlotinib, brain metastases, non‐small cell lung cancer, perilesional edema, stereotactic radiosurgery

## Abstract

**Introduction:**

About 50% of patients with non‐small cell lung cancers (NSCLC) are diagnosed with brain metastases during treatment, and stereotactic radiosurgery (SRS) is an important treatment for brain oligometastasis. Some patients with brain metastases have cerebral edema before treatment, and radiation therapy may also cause, or aggravate brain edema. Vascular endothelial growth factor (VEGF) promotes angiogenesis and increase vascular permeability, and previous studies have shown that anti‐VEGF treatment can reduce brain edema. We hypothesized that anlotinib hydrochloride can reduce perilesional edema around brain metastases, create conditions for subsequent SRS, increase local control rate and improve patient prognosis.

**Methods:**

From one week before stereotactic radiosurgery, patients begin to receive anlotinib once a day (12 mg) from day 1–14 of a 21 day cycle, with two cycles in total. Brain magnetic resonance imaging (MRI) scan is taken before treatment, one week and one month after medication. A total of 50 patients will be included in this study. The primary endpoint is the Edema Index, and the secondary endpoints are intracranial objective response rate (iORR), intracranial progression‐free survival (iPFS), objective response rate (ORR), disease control rate (DCR), progression‐free survival (PFS), overall survival (OS), safety, and the rate of SRS after anlotinib treatment.

**Discussion:**

This study is a multicenter, prospective, single‐arm, phase II clinical study, and explores the efficacy and tolerability of SRS with anlotinib in NSCLC patients with limited brain metastases. The aim of the study is to provide new treatment options for NSCLC patients with brain metastases.

## Introduction

Brain metastases are the most common malignant intracranial tumors. The incidence of brain metastases is about 40% in all patients with malignant tumors, of which 50% occur in lung cancer.^1^ With the development of targeted therapy, immunotherapy, and radiation therapy, the survival time of lung cancer patients continues to lengthen, but the treatment of brain metastases is still difficult in lung cancer treatment.^2^ For brain metastases from lung cancer, radiation therapy is an important therapeutic approach.^3^, ^4^ Stereotactic radiosurgery for the treatment of brain metastases can lead to higher local control rates and lower radiation doses to surrounding normal brain tissue, which plays an important role in the treatment of brain metastases. However, for patients with obvious cerebral edema, stereotactic radiosurgery may induce or aggravate cerebral edema,^5^ which cause poor tolerance to this treatment. Hence, it is necessary to pretreat edema before treatment with stereotactic radiosurgery (SRS). Unfortunately, traditional treatment, such as mannitol and hormones, is less effective in some patients with refractory edema.

The article "Stereotactic radiosurgery combined with anlotinib for limited brain metastases with perilesional edema in non‐small cell lung cancer: Rvision‐001 study protocol" was published in 2020. Journal: Thorac Cancer.

Vascular endothelial growth factor (VEGF) promotes angiogenesis and increases vascular permeability, and antiangiogenic drugs theoretically have the effect of reducing cerebral edema.^6^, ^7^ Anlotinib is a multitargeted tyrosine kinase receptor inhibitor, especially for vascular endothelial cell growth factor receptor 2 (VEGFR2) and VEGFR3,^8^ and is approved for third‐line treatment of non‐small cell lung cancer (NSCLC).^9^, ^10^ For patients with brain metastases accompanied by cerebral edema, anlotinib can reduce the permeability of blood vessels through antiangiogenesis, and theoretically reduce brain edema and enhance the effect of radiosurgery.

Based on this information, we planned a phase II study of stereotactic radiosurgery with anlotinib for limited brain metastases with perilesional edema in NSCLC. Here, we introduce the details of this study.

## Protocol of study revision‐001

### Objectives

This study aims to explore the efficacy and the tolerability of stereotactic radiosurgery with anlotinib for limited brain metastases with perilesional edema in NSCLC.

### Study design

This is a single‐arm, prospective, phase II study. An overview is shown in Fig 1.

**Figure 1:** Rvision‐001 study design. DCR, disease control rate; iORR, intracranial ORR; iPFS, intracranial PFS; ORR, objective response rate; OS, overall survival; PD, disease progression; PFS, progression‐free survival; SRS, stereotactic radiosurgery.

### Endpoints

The primary endpoint is the Edema Index. The “Edema Index (EI)” is calculated per the equation of “edema index = (perilesional edema volume)/tumor volume. All volume calculations are made on MRI by integration of the areas over a contiguous set of axial slices. The perilesional edema is defined on T2‐weighted sequences. The gross tumor volume is defined on T1 gadolinium‐enhanced images. Secondary endpoints are intracranial objective response rate (iORR), intracranial progression‐free survival (iPFS), objective response rate (ORR), disease control rate (DCR), progression‐free survival (PFS), overall survival (OS), safety and the rate of SRS after anlotinib treatment.

The article "Stereotactic radiosurgery combined with anlotinib for limited brain metastases with perilesional edema in non‐small cell lung cancer: Rvision‐001 study protocol" was published in 2020. Journal: Thorac Cancer.

## Key eligibility criteria

### Inclusion criteria

Patients must fulfill all the following criteria: (i) patients voluntarily participate in this study, with their signed informed consent; (ii) patients must be pathologically diagnosed with NSCLC, with brain metastases and measurable lesions; (iii) patients are aged between 18–80 years; with expected survival time > 3 months; (iv) patients have no more than five brain metastases; (v) patients with normal organ function within seven days prior to treatment, and (vi) female patients should agree to use contraceptives during and within six months after the study.

The following criteria must also be met: (a) blood routine examination criteria: (i) hemoglobin (HB) ≥90 g/L; (ii) absolute neutrophil count (ANC) ≥1.5 ×10^9^/L; (iii) platelet (PLT) ≥80 × 10^9^/L. (b) Biochemical tests must meet the following criteria: (i) total bilirubin (TBIL) ≤1.5 times of upper limit of normal (ULN); (ii) alanine aminotransferase (ALT) and aspartate aminotransferase (AST) ≤2.5 ULN, if liver metastasis occurred, ALT and AST ≤5 ULN, and (iii) serum creatinine (Cr) ≤1.5 ULN or creatinine clearance (CCr) ≥60 mL/min.

### Exclusion criteria

Patients are excluded from the study if they meet any of the following criteria: (i) patients who had previously used antiangiogenic agents within one month; (ii) patients with small cell lung cancer (including small cell carcinoma and non‐small cell carcinoma mixed lung cancer); (iii) patients with lung squamous cell carcinoma that involved pulmonary hilar, or NSCLC with hemoptysis; (iv) patients with cerebral infarction and cerebral hemorrhage; (v) patients without perilesional edema; (vi) patients with more than grade two (NCI‐CTCAE v4.0) acute toxicity reaction due to any previous treatment; (vii) patients with difficulty to take oral medication, such as dysphagia, chronic diarrhea and intestinal obstruction, etc; (viii) patients with visceral dissemination and severe symptoms, which could cause death in a short period; (ix) patients with any severe and/or uncontrolled disease; (x) patients received a major surgical treatment, biopsy or significant traumatic injury within one month; (xi) patients with any signs or medical history of bleeding, unhealed wounds, ulcers or fractures; (xii) patients underwent artery/venous thrombotic events with two months, such as deep vein thrombosis and pulmonary embolism; (xiii) patients with a history of psychotropic medicine abuse and cannot quit or have mental disorders; (xiv) patients were diagnosed with disease which will severely endanger their security and influence the completion of this research, and (xv) patients who still can't tolerate SRS after anlotinib treatment, even after adding mannitol, and have to receive steroid treatment.

The article "Stereotactic radiosurgery combined with anlotinib for limited brain metastases with perilesional edema in non‐small cell lung cancer: Rvision‐001 study protocol" was published in 2020. Journal: Thorac Cancer.

### Treatment plan

Treatment consists of anlotinib monotherapy plus SRS for brain metastases. Anlotinib is administered 12 mg/day from one week before the MRI‐based simulation, day 1–14 of a 21 day cycle, two cycles in total. SRS for brain metastases is delivered using CyberKnife (CK) system. The target volume is identified using a CT and enhanced MRI image fusion. The gross tumor volume (GTV) is delineated on the T1 gadolinium‐enhanced sequences. An isotropic margin of 1.25/1.6 mm is added around GTV to obtain the planning target volume (PTV). The SRS prescription doses are chosen according to the routine treatment of participating institutions.

### Follow‐up and assessment

To assess the efficacy, brain MRI is taken one month after SRS, and every three months after that. The Edema Index will be calculated based on the MRI at the time of simulation and one month after SRS. The cerebral edema symptoms, dehydration treatment (glucocorticoids and mannitol) will be recorded and quality of life will be evaluated by the EORTC QLQ‐BN20. Adverse events are graded using the Common Terminology Criteria for Adverse Events, version 4.0.

### Statistical design

In this study, the brain edema index was used as the main efficacy index to estimate the sample size. With reference to the relevant data of the antiangiogenic drug bevacizumab for the treatment of cerebral edema,^7^ the self‐control before and after treatment: the cerebral edema index before treatment was 15.51 ± 7.10, the cerebral edema index after treatment was 9.02 ± 4.40, and the difference between the cerebral edema index before and after treatment was 6.49. The combined standard deviation is seven, the one‐sided test level α is 0.05, and the statistical power of 0.90. According to the formula: n = (z_1−α/2_ + z_1−β_)^2^S^2^/δ^2^, 40 patients will be enrolled. Although bevacizumab and anlotinib are all antiangiogenic drugs, the action mechanisms are not exactly the same. Meanwhile, the uncertainty of tests such as shedding rate of 20% are considered, and the sample size is expanded to 50.

### Ethical considerations

The protocol was approved by the institutional review board of each participating institution. Written informed consent is obtained from all participants before any screening or inclusion procedures. This protocol was registered at the website of http://clinicaltrials.gov (protocol identification number NCT04147728). The results will be published in a peer‐reviewed journal.

The article "Stereotactic radiosurgery combined with anlotinib for limited brain metastases with perilesional edema in non‐small cell lung cancer: Rvision‐001 study protocol" was published in 2020. Journal: Thorac Cancer.

## Discussion

Revision‐001 is a multicenter, single‐arm, phase II clinical study, and aims to explore the efficacy and the tolerability of stereotactic radiosurgery with anlotinib for limited brain metastases with perilesional edema in NSCLC. SRS is widely used in the treatment of brain oligometastases of NSCLC. However, SRS can aggravate or induce perilesional edema. VEGF promotes angiogenesis and vascular permeability, and thus plays an important role in cerebral edema. Anti‐VEGF treatment could theoretically reduce brain edema and potentially improve efficacy of SRS.

Anlotinib is an orally administered multitarget tyrosine kinase inhibitor for tumor angiogenesis and proliferative signaling, which targets receptor tyrosine kinases VEGFR1/2/3, epidermal growth factor receptor (EGFR), fibroblast growth factor receptor 1 to 4, platelet‐derived growth, factor receptor α and β, and stem cell factor receptor. The advantages of combination anlotinib and stereotactic radiosurgery are as follows: (i) anlotinib can regulate permeability of blood vessels and thus reduce perilesional edema, which allows better tolerance to stereotactic radiotherapy; (ii) anlotinib probably enhances the efficacy of radiosurgery. Anlotinib can promote the normalization of blood vessels and increase the oxygenation of tumor tissues, thereby increasing the efficacy of radiosurgery. In addition, studies have proved that anlotinib itself can prolong OS and PFS in patients with NSCLC cancer,^11^ and (iii) previous studies have shown that other antiangiogenic drugs, such as bevacizumab, and endostar, have the effect of reducing cerebral edema. However, there is a lack of high‐level research evidence. Furthermore, these two drugs are intravenous, while anlotinib is an orally administered drug, which is more convenient for patients undergoing stereotactic radiosurgery in outpatients.

This study has limitations. First, the sample size of this study is relatively small. However, due to the lack of previous safety data of anlotinib combined with stereotactic radiosurgery for cerebral edema, a smaller sample size is more suitable. Second, although anlotinib is only approved for third or more lines of systemic treatment in patients with advanced NSCLC, the inclusion criteria of this study did not restrict the history of first‐line /second‐line/third‐line treatment, which may lead to greater heterogeneity of the patients in the previous treatment history. However, in clinical practice, stereotactic radiosurgery may be necessary for most patients with brain oligometastasis, regardless their treatment history. Furthermore, the main endpoint of this study is the Edema Index, which is probably not affected by previous antitumor treatments except antiangiogenic agents.

The article "Stereotactic radiosurgery combined with anlotinib for limited brain metastases with perilesional edema in non‐small cell lung cancer: Rvision‐001 study protocol" was published in 2020. Journal: Thorac Cancer.

This is the first study to explore the efficacy and tolerability of SRS with anlotinib in NSCLC patients with limited brain metastases. We believe that the results of this study will provide new treatment options for NSCLC patients with brain metastases.

## Disclosure

The authors confirm that there is no conflict of interest.
